The article "Analysis of Risk Factors of Neurobiological Pipeline Care and Investigation of Preventive Measures" was retracted in 2023. Reasons: signs of a paper mill; suspected computer-generated content; unreliable results or conclusions; lack of ethics approval or compliance.

# Analysis of Risk Factors of Neurobiological Pipeline Care and Investigation of Preventive Measures

**DOI:** 10.1155/2021/3572265

**Published:** 2021-10-13

**Authors:** Lin Sun, Qian Wang, Jinzhi Feng

**Affiliations:** Department of Neurosurgery, Xiangyang Central Hospital, Affiliated Hospital of Hubei University of Arts and Science, Xiangyang, Hubei 441021, China

## Abstract

During clinical care, most neurosurgical patients are critically ill. They have sudden onset of illness that should be treated on time with proper care. The patients require continuous hospitalization for proper treatment. The recovery of patients may be relatively slow and takes some time. *Patients and Methods*. To explore where the risks of pipeline care lie and the preventive measures. (1) In this paper, 100 neurosurgical patients were treated in our hospital from September 2018 to March 2020. They were firstly selected and divided into two groups. Group A was implemented with routine pipeline care and group B was implemented with the intervention developed by the pipeline team. (2) The design and SMOTE assume that, during the generation of a new synthetic sample of minority classes, the immediate neighbors of the minority class instances were also all minority classes, regardless of their true distribution characteristics, to analyze risk factors during care and summarize preventive measures. *Results*. The experimental results showed that the total efficiency of nursing care was higher in group B as compared to group A, *P* < 0.05; also, the number of pipeline accidents was lower in group B. *Conclusion* It is important to be meticulous and thoughtful in pipeline care and to comprehensively analyze the possible risk events and then propose preventive measures so that risk events can be reduced.

## 1. Introduction

In clinical care, most patients in neurosurgery are critically ill or have a sudden onset of illness. Many patients require continuous hospitalization for some time and have a relatively slow recovery rate. Under such circumstances, the psychological state of patients is often subject to great fluctuations, and nursing staff may face risks in all aspects of care [1]. At the same time, with the improvement of living standards, people's awareness of their rights has also increased, which has led to more and more nursing disputes in hospitals. In the actual nursing process, neurological nursing risk factors can be summarized into the following aspects [2]:

- Responsibility awareness factor
- Nursing technology factor
- Nurse-patient communication factor
- Patient psychological factor

The details of these aspects in the context of nursing risk factors are given as follows.

### 1.1. Rising the Risk Awareness of Nursing Staff

(1) To better control the risk factors in neurological care, strict risk management measures need to be developed first, to establish an active precautionary system to avoid various risk incidents. To achieve this goal, nursing staff need to raise their risk awareness and identify risk factors and safety hazards promptly. Also, they need to take scientific measures to address them [3]. To this end, hospitals need to provide regular training to help nursing staff recognize the importance of safety awareness in the nursing process. In addition, hospitals need to develop a management plan that meets the needs of neurological care, taking into account the special characteristics of neurosurgery. To avoid the occurrence of various risk events, it needs to be supervised by a dedicated person.
(2) By collecting, summarizing, and analyzing massive data information and precisely exploring the invisible knowledge contained in it, the value of data information can be fully revealed after deep mining of medical big data, which can provide a great impetus to medical research and clinical care [4]. For patient groups, good medical big data can help them get a better treatment experience and effectively avoid excessive economic investment. For the development of modern medical research, its application can provide good help for future pharmaceutical research and development, clinical care, and disease diagnosis [5]. At the same time, the deep and clear excavation and analysis of the public's medical big data can effectively realize the supervision and monitoring of people's health conditions, to distinguish patients with high-risk diseases, which has a great influence on the actual development of diseases [6]. The effective analysis and application of medical big data technology absolutely cannot be separated from the support of complete data mining technology. Along with the progress and development of modern science and technology, the development of data mining technology has become more and more perfect and specific, and the research direction has been significantly broadened. The application of data mining technology in medical big data is mainly reflected in the following points:
  - Association rule mining.
  - Followed by anomaly mining.
  - Derivation of a large number of new algorithms. Such algorithms will for the analysis of medical big data applications; thereafter these algorithms will provide a solid support role for the subsequent analysis and application of medical big data and are the basis for creating a medical big data system [7, 8].
(3) Communication is an important part of nursing. Therefore the development of a positive nurse-patient relationship is essential for the delivery of quality nursing care.
(4) Patient psychological factor also plays an essential role in physical illness. The psychological factors might influence the immunity and immune system of a patient. Therefore it is required to understand the psychological condition of patients.

### 1.2. Preventive Measures

Neurosurgical patients often receive drainage tubes. They are at risk for total or partial dislodgement, excessive drainage, and obstruction or entrapment during tube care. These patients are often comatose and aphasic, which can lead to exacerbation or even death if not properly managed [9]. Therefore, it is important to identify risk factors during tubing care and take targeted preventive measures.

Following are the major contributions of this paper:

1. This paper proposes the correct evaluation of classification performance for selecting classification features and classifier parameters. We use the *F*-measure and AUC evaluation criteria instead of the traditional method based on classification accuracy.
2. The SMOTEC algorithm has used the modified SMOTE method to oversample a small number of class instances in the training dataset to increase the number of minority class samples compared to the SVM feature to design a clustering algorithm to clean the data set after oversampling.
3. An improved SMOTE and clustering-based method are used to process the unbalanced dataset, and then SMO is used to construct the classification plan and make predictions and the pseudocode of the SMOTEC-SMO algorithm. The design and SMOTE assumed that the immediate neighbors of the minority class instances were also all minority classes in the process of generating a new minority class composite sample, without considering their true distribution characteristics, analyzing the risk factors during care, and summarizing preventive measures.
4. The experiments, statistical analysis, and results showed that the total efficiency of care was higher in group B compared with the group A, *P* < 0.05; also, the number of pipeline accidents was lower in group B.

The outline of this paper is given below:

In Section 2 we discussed the performance evaluation of unbalanced classification.

In Section 3 we discussed the proposed methods: SMOTE-Clustering SMO algorithm, clustering-based example undersampling method, and SMOTEC-SMO algorithm descriptions are discussed.

In Section 4 we discussed simulation experiments; general information of the patients on which experiments were carried out, methods, observed indicators, and statistical analysis for different experiments are discussed.

In Section 5 different data obtained during experiments are compared with the following four online learning approaches for further results. It includes UCB1, HOO, LinUCB, and ACR.

In Section 6 of clustering analysis results, the comparison of effective efficiency of nursing and pipeline incidents is discussed below in this section.

## 2. Related Work

This section shows the correct evaluation of unbalanced data classification for selecting classification features and classifier parameters.

### 2.1. Performance Evaluation of Unbalanced Data Classification

The correct evaluation of classification performance is an important guide for selecting classification features and classifier parameters. To evaluate the performance of classifiers for unbalanced data sets, we should focus on the classification of a small number of samples. In this paper, we use the F-measure and AUC evaluation criteria instead of the traditional method based on classification accuracy [10].

Table 1 shows the confusion matrix for the two-class classification problem, which is a common method to evaluate the classification performance of algorithms in the field of machine learning. TP and TN indicate the number of correctly classified majority and minority classes, respectively, while FN and FP indicate the number of disqualified minority and majority classes, respectively [10].

The confusion matrix leads to two important concepts: Recall and Precision, as shown in equation (1):

(1) $$\begin{array}{c} \text{True positive rate}\left(\text{TPR},{\text{Acc}}^{+}\right)=\frac{\text{TP}}{\text{TP}+\text{FN}}=\text{Recall},\\ \text{Positive predictive value}=\frac{\text{TP}}{\text{TP}+\text{FP}}=\text{Precision}. \end{array}$$

The *F*-measure is a classification evaluation indicator that takes into account both accuracy and completeness. *β* is the parameter used to adjust the relative importance of accuracy and completeness and is calculated as shown in

(2) $$\begin{array}{c} F-\text{measure }=\frac{\left(1+\beta^{2}\right)\times \text{Precision}\times \text{Recall}}{\beta^{2}\text{Precision}+\text{Recall}}\times 100\%, \end{array}$$

where *β* takes the values [0, ∞]. When 0 < *β* < +∞, *F*_*B*_ there is a compromise between Precision and Recall. *β*=0, *F*_*B*_=Precision, *β*=*∞F*_*B*_=Recall, and *β* < 1 emphasizes the role of Precision; *β* > 1 emphasizes the role of Recall. In most experiments, the *F*1 metric is used; that is, *β* takes a value of 1. In this case, Precision and Recall are equally important in evaluating the performance of the algorithm, and their weights are equal. When *β* = 1, we can simplify equation (2) to equation (3), where *F*1 represents the summed average of the accuracy rate and the recall rate.

(3) $$\begin{array}{c} F_{1}=\frac{2\times \text{Precision}\times \text{Recall }}{\text{ Precision}+\text{Recall }}=\frac{2}{\left(1/\text{Precision}\right)+\left(1/\text{Recall}\right)}. \end{array}$$

The summed mean of the two values is often close to the smaller of the two values. Only when both the full rate and the accuracy rate are high can we ensure a high *F*-measure value. The *F*-measure is a valid evaluation criterion for the classification problem of unbalanced data sets to correctly evaluate the classification performance of the classifier for each class.

## 3. Proposed Method

In this section, the method used using SMOTE-Clustering SMO algorithm, clustering-based example undersampling method, and SMOTEC-SMO algorithm descriptions are discussed.

### 3.1. SMOTE-Clustering (SMOTEC) SMO Algorithm

The SMOTEC algorithm [11] first uses the modified SMOTE (synthetic minority oversampling technique) method to oversample a small number of class instances in the training dataset to increase the number of minority class samples. Then it uses the SVM feature to design a clustering algorithm to clean the data set after oversampling. Redundant or noisy data samples are removed. By oversampling and cleaning the original dataset, some useful samples are retained, which reduces the size of the dataset and enhances the efficiency of the SMO training implementation.

### 3.2. Oversampling Method Is Based on the Improved SMOTE Idea

The SMOTE method assumes that the nearest neighbors of the minority class instances are also all minority classes in the process of generating new synthetic samples of minority classes and does not consider their real distribution characteristics. There is certain blindness in the nearest neighbor selection strategy, and the SMOTE algorithm can only recreate the interpolation of new synthetic samples for numerical data. To solve the problems of SMOTE method, we improve it: (1) according to the real distribution characteristics of different sample sets, (2) we choose to adjust the nearest neighbors of the minority class, (3) allow some samples of the majority class that are closer to the minority class to participate in the process of generating new samples, (4) remove the minority class samples that are farther away and, (5) adopt different generation methods for different cases of nearest neighbors. The objective is to control the nearest neighbor area of minority samples and improve the quality of synthetic samples [12].

Figure 1 shows the original unbalanced dataset, the five minority class nearest neighbors and five major class nearest neighbors of minority class sample *x*_1_ are {*x*_2_, *x*_3_, *x*_4_, *x*_5_, *x*_6_, *y*_1_, *y*_2_, *y*_3_, *y*_4_, *y*_5_}, among which three minority class nearest neighbors are {*x*_2_, *x*_3_, *x*_4_} and two major class nearest neighbors are {*y*_1_, *y*_2_}. *x*_5_, *x*_6_ is excluded from the candidate set of nearest neighbors because it is far from the minority class sample *x*_1_, and the majority class nearest neighbor *y*_1_, *y*_2_ is used to replace *x*_5_, *x*_6_ so that the five candidates nearest neighbors of *x*_1_ are determined to be {*x*_2_, *x*_3_, *x*_4_, *y*_1_, *y*_2_}. After that, new minority class composite samples are generated for each candidate nearest neighbor. SMOTE-NC and SMOTE-N methods are used to generate new composite minority class instances according to the different properties. In contrast to the numerical genus, there are two cases: (1) if the candidate nearest neighbor *x*_1_ is a minority class sample, the random number is rand [0, 1]; (2) if the candidate nearest neighbor of *x*_1_ is a majority class sample, the random number is rand [0, 0.5], which can control the newly generated synthetic samples to be as close as possible to the minority class instances and better avoid the occurrence of sample overlap. The results after the new samples are generated are shown in Figure 1(b). From Figure 1(b) it can be seen that the newly added minority class synthetic samples *x*_1_ are mostly distributed around them, basically maintaining the distribution of the original samples.

### 3.3. Clustering-Based Example Undersampling Method

Most undersampling techniques aim to balance the two classes of samples by reducing the number of majority class instances, but when the oversampling expansion multiplier is set too large, the minority class instances may also become majority class instances and the newly generated samples may not satisfy the data distribution. In this case, we devise a new data cleaning method that does not only undersample the most class instances but also performs a certain degree of data cleaning on both classes of sample data [13].

We first cluster the oversampled training set into multiple clusters *A*, *B*,…, *F* (as shown in Figure 2). As before, the “●” in the figure represents the majority class samples and the “★” represents the minority class samples. The classification plan of the support vector machine may pass through *C* and *D*; i.e., the support vectors may be generated in *C* and *D*, so all samples within them are retained. If all the samples within a cluster belong to the same class of instances, we will remove redundant data or wild points from it. Here, taking cluster *C* as an example, the steps are as follows.

1. Determine the magnitude of the similarity threshold in the range of (0, 1).
2. Calculate the mean sample $\bar{x}$ in cluster *C* according to the formula $\bar{x}=1/n_{i}\sum_{j=1}^{n_{i}}x_{j}$.
3. Find a point ${\bar{x}}_{c}$ ∈ *C* closest to $\bar{x}$ the cluster center.
4. Calculate the similarities *S*_*ic*_ and *S*_*ic*_ between each sample *x*_*i*_ ∈ *c* and ${\bar{x}}_{c}$ in cluster *C* [9]. If *s*_*ij*_ is greater than the similarity threshold, *x*_*i*_ is removed from cluster *C*; otherwise, it is reserved. The smaller the similarity threshold, the more simple the instances are removed. Among them, $\bar{x}$ is the center in the cluster, which is the number of samples in cluster *I*, *s*_*ij*_ represents the similarity between samples *x*_*j*_ and *x*_*i*_, and *x*_*k*_ represents the *k*-th attribute of the sample *x*_*ij*_.

### 3.4. SMOTEC-SMO Algorithm Descriptions

In this paper, an improved SMOTE and clustering-based method are used to process the unbalanced dataset. Then SMO is used to construct the classification plan and make predictions. Pseudocode of the SMOTEC-SMO algorithm is given below in Table 2.

## 4. Simulation Experiments

In this section, general information of the patients on which experiments were carried out, methods, observed indicators, and statistical analysis for different experiments are discussed.

### 4.1. General Information

A total of 100 neurological patients were selected for the study. 27 of these patients suffered from psychiatric disorders, 29 from aphasia, 13 from a coma, and 31 from emotional disturbance. Group A consisted of 27 males and 23 females, aged 29 to 75 years, with a mean of (52.94 ± 3.67) years; group B consisted of 28 males and 22 females, aged 30 to 76 years, with a mean of (53.11 ± 3.85) years. There was no significant difference in general information between the two groups, *P* > 0.05.

### 4.2. Methods

In group A, routine tube care was performed: (1) the nursing staff recorded the length of the tube, marked the tube uniformly and indicated the name of the tube, and fixed the tube with the help of satin tape; (2) patients who received an artificial airway were actively forced to drain the sputum, and for patients without a machine, the air outlet was covered with wet gauze to ensure the wetting of the airway; (3) inform the family of the importance of postoperative tubing and restrain the agitated patient with a restraining belt. In group B, the pipeline intervention measures were developed by the pipeline team: (1) set up a pipeline record sheet and a pipeline risk assessment sheet, through which the importance of pipeline marking and the color of the required marking were reasonably specified. The drainage was recorded uniformly, and the different pipelines were fixed secondarily with the help of 3 M tape; (2) give a “T” tube or an artificial nose to those who did not have an artificial airway with a machine and fix them with a “T” tube”; (3) establish a preoperative visit system, provide patients with leaflets, and introduce safety knowledge of tube protection to patients before and after surgery with the help of illustrated PPTs [14]; (4) formulate restraint assessment methods and adopt corresponding restraint methods through assessment of scores.

### 4.3. Observed Indicators

The observed indicators in the experiments are (i) total efficiency of care; (ii) pipeline accidents.

### 4.4. Judgment Criteria

Two groups according to their stability and degree of risk were identified during treatment: (1) ineffective: signs were unstable or excessive risk occurred during treatment; (2) effective: signs were generally stable and the degree of risk was mild.

### 4.5. Statistical Analysis

The data were compared with SPSS22.0 statistical software, and the count data were expressed as % (percentage), and *P* < 0.05 means significant difference [15].

Neurosurgical pipeline care exhibits different learning characteristics and their behavioral differences make their neurobiological pipeline care risk factors, preferences, and learning outcomes different from each other. Combining neurobiological pipeline care data and using different clustering algorithms to cluster learners into relatively homogeneous groups facilitate the prediction of behavioral characteristics and learning styles during the learning process. It can also facilitate the development of risk factors in neurological pipeline care [16].

For better observation, the collected neurobiological pipeline care is displayed as a scatter plot. The histograms are used to show the distribution of neurological pipeline care data, as shown in Figures 3 and 4, respectively.

The behavior of neurobiological pipeline care can be seen in two charts. The scatter plot shows a largely positive correlation between neurological pipeline care risk factors. The histogram shows nearly 300 risk factors for viewing neurobiological pipeline care, but nearly 100 for not viewing the video.

## 5. Experiments

Different data obtained during experiments are compared with the following four online learning approaches for further results. It includes UCB1, HOO, LinUCB, and ACR.

### 5.1. Benchmarking Scheme

We compared the approach in this paper with four comparable online learning approaches without privacy techniques.

  UCB1 [15]: classical bandits algorithm for solving E&P challenges without big data support and contextual information.
  HOO [17]: the X-arms bandits algorithm can support large data scenarios but does not consider the context.
  LinUCB [10]: a context-aware bandit algorithm that supports complex contexts.
  ACR [18]: a CMAB-based algorithm that utilizes a bottom-up tree structure and fixed clusters of services.

### 5.2. Results

The performance of the algorithms was evaluated by cumulative and average regret. In the experiments, various algorithms were run in the time range of 1 to 100000.

In Figure 5, we know that the cumulative regret of DCPT grows more slowly as the risk factors for neurological pipeline care increase. The results show that our method has less regret of only 21.98%, compared to 30.22%, 58.63%, and 72.66% for the other schemes, respectively. While the average regret of DCPT in Figure 6 decreases with the increase of rounds, especially in the first 1000 rounds, DCPT's regret decreases quickly and converges to the optimal strategy faster than the other algorithms. Meanwhile, LinUCB and ACR outperform UCB1 and HOO because they both consider the user's context, which is very important in the service selection process.

We also compared the results with other algorithms when the number of neurological pipeline care services was increased. As shown in Figures 7 and 8, the results indicate that DCPT outperforms the other methods. Since DCPT has a tree structure rather than bottom-up as in ACR, we have a good partitioning of *S* and outperformed other algorithms, indicating that DCPT can handle increasing datasets.

To more fully verify the performance effectiveness of the algorithm in this paper, we can vary the dimensions of the service space *d*_*s*_ and the context space *d*_*c*_ to evaluate the effectiveness of the spatial dimensions. As shown in Figures 9 and 10, a small amount of dimensionality leads to an increase in cumulative regret due to not considering enough information. We must consider the appropriate service dimension and context space. We ran DCPT using different privacy levels (*ϵ* Values). For the neurobiological pipeline care risk factor, to demonstrate the trade-off between service selection accuracy and privacy levels, we set *ϵ* = 0.01, 0.05, 0.5, 1 and compared the performance with the no-privacy condition.

## 6. Clustering Analysis Results

The comparison of effective efficiency of nursing and pipeline incidents is discussed below in this section.

### 6.1. Comparison of Nursing Outcomes

Compared with group A, the total efficiency of care was higher in group B, up to 96.00%, *P* < 0.05, as shown in Table 3.

### 6.2. Comparison of Pipeline Accidents

There were three cases of accidental tube events in group A, one of which was catheter dislodgement and the remaining two cases were obstruction of the tracheal tube, as shown in Table 4.

There was only 1 unexpected event in group B, which was tracheal tube obstruction, as shown in Table 5.

### 6.3. Discussion

There are many risk factors in pipeline care, as follows:

1. lack of nursing staff awareness of pipeline management risks: The work of ward treatment and care is more complicated, and nurses with lower seniority do not have enough experience, risk awareness, judgment, and resilience. They are unable to make an accurate assessment of the patient's condition. When the patient has an obstruction or a detached pipeline, it is difficult to detect and do a good job in time. Therefore, the condition can be aggravated [2].
2. Pipeline factors: (i) problems with the pipeline itself, such as the pipeline not being marked with a scale or the scale not being marked, can lead to pipeline care risks; (ii) problems with the method of fixing the pipeline: Some patients need to receive cephalothorax drainage, and when nurses fix the pipeline by wrapping sutures and leading them out to the dressing site, the patient's position often changes. This leads the scalp not adhering well to the tape, which can easily displace or loosen the fixation tape, failing to fix firmly [3]. In addition, the orchotomy tether may loosen due to swallowing and violent coughing, forcing the tracheal tube out when pulling on the ventilator tube.
3. Other factors: Sutures may break due to age when they are fixed for a long time or impregnated with ooze for a long time.
4. Environmental factors: Unsuitable temperature and humidity in the ward will affect the patient's breathing, which will make patients receiving an artificial airway more prone to respiratory distress.
5. The ward is quiet at night, so when the alarm generated by the instrument is too loud, it will frighten the patient, which will cause the risk of unplanned excitation [4].
6. Patient factors: Most patients have a brain injury and lack of self-control, and their consciousness needs to be observed because their condition is easy to change, so they cannot be provided with excessive sedation during treatment. When the patient is agitated, the tube will fall off and aggravate their condition. Some patients are sometimes awake and sometimes fuzzy, and when their consciousness is fuzzy, they will withdraw the tube by themselves.
7. Family members: Some family members lack knowledge and do not listen to the nurses' advice. They sometimes remove the patient's fixation belt or restraint material without understanding, which can greatly increase the risk of catheterization.

For pipeline care, the following preventive measures can be taken:

1. Establish a management group: (i) Organize risk education for nurses: The adequacy of nurses' risk awareness not only affects the quality of care but also determines the attitude toward care. At the time of admission, the team members provide pipeline safety education to new nurses to help them pay more attention to the importance of pipeline care with the help of warning cases. The nursing quality control office will establish a high-risk risk assessment form: a score will be set for each pipeline situation, and the score will be positively correlated with the risk level, and the risk of the pipeline will be clarified by superimposing each score, to encourage the responsible nurses to pay more attention to the management of nursing care.
2. Improvement of catheter care: (i) Development of a manual of knowledge of drainage tubes: The manual is used by junior nurses to learn about catheters to help them improve their professionalism and to consult strategies when problems arise during care. (ii) Develop a catheter record sheet: Use the record sheet to record catheter placement, medication changes, and removal time for better management.
3. Do a good job of artificial airway care: (i) reasonably adjust the room temperature and humidity; (ii) provide nurses with nursing training; (iii) equip those who receive an artificial airway ventilator with a humidifier to do a good job of heating and humidifying and may take artificial airway nebulization measures; (iv) adopt a “T” tube or artificial nose and heating and humidifying for those who do not receive a ventilator [5].
4. Nurses should strictly implement medical advice: the degree of implementation of medical advice by nurses influences the chance of risk, and only by strictly implementing medical advice can patients receive reasonable treatment.
5. Communicate well with patients' families: (i) improve the visit system and establish a visit leaflet before surgery and introduce the role of different tubes for patients and their families with the help of illustrated PPTs; (ii) communicate with patients promptly after surgery to prevent their negative psychology, to eliminate patients' excessive behavior and reduce the possibility of tube risks.

In summary, inadequate management of neurological care can easily lead to risk events such as blockage or dislodgement of the tube. It can not only threaten the patient's treatment but even affect life safety in serious cases. Therefore it must be taken seriously. The risk factors of pipeline care are many, involving more factors such as nurses' awareness, patients themselves, pipeline quality, and the environment. The nursing staff must always be alert to the importance of preventing pipeline risks and strive to do a good job in all aspects of care.

## 7. Conclusions

In the process of clinical treatment, most patients in neurosurgery belong to patients with more critical conditions or sudden onset of illness. Many of them need to be continuously hospitalized for a while to receive treatment, while their recovery rate is relatively slow. This paper was designed with SMOTE in the process of generating a new minority class synthetic sample assuming that the immediate neighbors of the minority class instances are also all minority classes. Their real distribution characteristics, analyzing the risk factors during care, and summarizing preventive measures were not considered. The experimental results showed that the total efficiency of neurobiological pipeline care was higher, *P* < 0.05 [19].

## Figures and Tables

**Figure 1:** Processing process of the improved SMOTE algorithm.

**Figure 2:** Schematic diagram of sample clustering.

**Figure 3:** Scatter plots of the relationship between risk factors for neurological pipeline care.

**Figure 4:** Histogram distribution of risk factors for neurological pipeline care.

**Figure 5:** Average regret.

**Figure 6:** Cumulative regret.

**Figure 7:** Cumulative regret.

**Figure 8:** Average regret.

**Figure 9:** Cumulative regret for different *d*_*s*_.

**Figure 10:** Cumulative regret for different letters of credit.

**Table 1:** Confusion matrix.

	Positive predicted	Negative predicted
Positive class	True positives (TP)	False negatives (FN)
Negative class	False positive (FP)	True negatives (TN)

**Table 2:** SMOTEC-SMO algorithm descriptions.

**Input**: Number of minority class samples *N*; the number of clusters *K*; similarity threshold *S*; SMOTE oversampling expansion multiplier *T*%.
**Output:** SMO classification plane and prediction results.
Initialize the hypermastigote, which include the number of iterations *t*, the learning rate *L*, the hypermastigote of the recurrent neural network *β*_1_, *β*_2_, and the computational gradient of the model *g*_*t*_;
(1) BEGIN/*∗* Improved SMOTE Over-sampling*∗*/
(2) *G* = int(*N* *∗* *T*%); //Oversampling a few class examples
(3) For *i* = 1 to *G*
(4) For *I* = 1 to *N*
(5) Compute k-NN *x*_*i*_; //Find 5 nearest neighbors of *x*_*i*_
(6) For *i* = 1 to nuberattr/∗nuberattrIndicates the number of attributes*∗*/
(7) If *x*_*ij*_ is a numeric attribute
(8) If if *x*_*ij*_ ∈ Minority then *x*_*nj*_=(*x*_*i*_ − *x*_*ki*_)^*∗*^
(9) Rand(1)//Different generation methods for different cases of near neighbors
(10) elseif if *x*_*ij*_ ∈ Minority then *x*_*nj*_=(*x*_*i*_ − *x*_*ki*_)^*∗*^
(11) ^∗^rand(0.5)
(12) endif
(13) endif
(14) endFor
(15) endFor
(16) endFor
(17) *k* − NN(*x*_*j*_, *x*_*j*_′)
(18) If *j* ∈ Minority then *x*_*nj*_=(*x*_*i*_ − *x*_*ki*_)^*∗*^, /*∗* If *j* is a continuous value *∗*/
(19) If *j* ∈ nominal then *δ*_*n*_∑_*j*=1_^*c*^|*N*_*j*_, *x*_*j*_, *c*/*N*_*j*_, *x* − *N*_*j*_, *x*_*j*_′, *c*/*N*_*j*_, *x*′|(VDM) If *J* is a discrete value Δ=*δ*_*c*_+*δ*_*n*_ / ^*∗∗∗*^ Clustering under-samping ^*∗∗∗*^/
(20) Clustering divides the training data set into *K* clusters;
/ ^*∗∗∗∗∗∗∗∗*^ SMO ^*∗∗∗∗∗∗*^/SMOTraining; //Training with sequential minimum optimization (SMO) algorithm
SMOProjections;
END

**Table 3:** Comparison table of effective efficiency [*n* (%)].

Classification	*n*	Invalid (example)	Effective (example)	Remarkable effect (example)	Total effective (cases)
Group A	50	8 (16.00)	20 (40.00)	22 (44.00)	42 (84.00)
Group B	50	2 (4.00)	24 (48.00)	24 (48.00)	38 (95.00)
*x* ^2^	—	—	—	—	4.114
*P*	—	—	—	—	<0.05

**Table 4:** Group A write pipeline incident.

Event name	Number of cases	Reason	Time	Consequence
Catheter prolapse	1	Prolapse with urine	At night	Urinary incontinence
Tracheal tube obstruction	2	Failure to suck sputum in time	day	Affect breathing

**Table 5:** Group B write pipeline incidents.

Event name	Number of cases	Reason	Time	Consequence
Tracheal tube obstruction	1	Incomplete sputum suction	Day	Formation of consciousness disorder

## Data Availability

The datasets used and analyzed during the current study are available from the corresponding author upon reasonable request.

## References

[1] Rosińczuk J., Kotuniuk A. (2015). Analysis of the causes of lumbar disc herniation in patients treated neurosurgical due to it. *The Journal of Neurological and Neurosurgical Nursing*.

[2] Morshed R. A., Young J. S., Safaee M. (2019). Delirium risk factors and associated outcomes in a neurosurgical cohort: a case-control study. *World neurosurgery*.

[3] Wang J., Ji Y., Wang N. (2018). Risk factors for the incidence of delirium in cerebrovascular patients in a Neurosurgery Intensive Care Unit: a prospective study. *Journal of Clinical Nursing*.

[4] Hussein K., Rabino G., Feder O. (2019). Risk factors for meningitis in neurosurgical patients with cerebrospinal fluid drains: prospective observational cohort study. *Acta Neurochirurgica*.

[5] Uche E. O., Mezue W. C., Ajuzieogu O. (2020). Improving capacity and access to neurosurgery in sub-Saharan Africa using a twinning paradigm pioneered by the Swedish African Neurosurgical Collaboration. *Acta Neurochirurgica*.

[6] Liu J., Gormley N., Dasenbrock H. H. (2019). Cost-benefit analysis of transitional care in neurosurgery. *Neurosurgery*.

[7] Yu X., Zhan D., Liu L., Lv H., Xu L., Du J. (2021). A privacy-preserving cross-domain healthcare wearables recommendation algorithm based on domain-dependent and domain-independent feature fusion. *IEEE Journal of Biomedical and Health Informatics*.

[8] Punchak M., Mukhopadhyay S., Sachdev S. (2018). Neurosurgical care: availability and access in low-income and middle-income countries. *World neurosurgery*.

[9] Kumar V. A. K, Sai N. K., Kumar V. A. (2019). The outcome analysis and complication rates of tracheostomy tube insertion in critically ill neurosurgical patients; a data mining study. *Bulletin of Emergency and Trauma*.

[10] Yu M., Jin J., Wang X., Yu X., Zhan D., Gao J. (2021). Development and design of flexible sensors used in pressure-monitoring sports pants for human knee joints. *IEEE Sensors Journal*.

[11] Xu Z., Shen D., Nie T., Kou Y., Yin N., Han X. (2021). A cluster-based oversampling algorithm combining SMOTE and k-means for imbalanced medical data. *Information Sciences*.

[12] Robertson F. C., Logsdon J. L., Dasenbrock H. H. (2017). Transitional care services: a quality and safety process improvement program in neurosurgery. *Journal of Neurosurgery*.

[13] Gaspari C. H., Lafayette S., Jaccoud A. C., Kurtz P., Lavradas L. A., Cavalcanti D. D. (2018). Safety and feasibility of out-of-bed mobilization for patients with external ventricular drains in a neurosurgical intensive care unit. *Journal of Acute Care Physical Therapy*.

[14] Zhang C., Xie T., Yang K. (2019). Positioning optimisation based on particle quality prediction in wireless sensor networks. *IET Networks*.

[15] Kingsberg S. A., Clayton A. H., Pfaus J. G. (2015). The female sexual response: current models, neurobiological underpinnings and agents currently approved or under investigation for the treatment of hypoactive sexual desire disorder. *CNS Drugs*.

[16] Schumann G., Loth E., Loth E. (2010). The IMAGEN study: reinforcement-related behaviour in normal brain function and psychopathology. *Molecular Psychiatry*.

[17] Froehlich T. E., Anixt J. S., Loe I. M., Chirdkiatgumchai V., Kuan L., Gilman R. C. (2011). Update on environmental risk factors for attention-deficit/hyperactivity disorder. *Current Psychiatry Reports*.

[18] Hwang G., Dabbs K., Conant L. (2019). Cognitive slowing and its underlying neurobiology in temporal lobe epilepsy. *Cortex*.

[19] Bekelis K., Missios S., MacKenzie T. A. (2018). Correlation of hospital magnet status with the quality of physicians performing neurosurgical procedures in New York State. *British Journal of Neurosurgery*.

